The article "The Clinical Features and Treatment Strategy of Parathyroid Cancer: A Retrospective Analysis" was published in 2022. Journal: Biomed Res Int.

# The Clinical Features and Treatment Strategy of Parathyroid Cancer: A Retrospective Analysis

**DOI:** 10.1155/2022/1913900

**Published:** 2022-09-23

**Authors:** Chen Wang, Kaixue Wen, Li Dai, Shuxin Wen, Yuhao Zhang

**Affiliations:** ENT Department, Third Hospital of Shanxi Medical University, Shanxi Bethune Hospital, Shanxi Academy of Medical Sciences, Tongji Shanxi Hospital, Taiyuan Shanxi 030032, China

## Abstract

**Objective:**

To review the features and treatment of parathyroid cancer in our series. Explore the suitable extent of initial surgery and the effect of adjuvant radiotherapy in local recurrence.

**Methods:**

Seven cases of parathyroid cancer presented from 2014 to 2021. The presenting features, diagnosis, and treatment are presented.

**Results:**

Only two patients had multiple manifestations of hypercalcemia. Marked hypercalcemia, which was revealed to be an average of 13.9 mg/dl (range from 11.8 mg/dl to 15.8 mg/dl), was observed in four patients (57%). The others' serum calcium levels were in the normal range with an average of 9.9 mg/dl (range from 8.6 mg/dl to 10.8 mg/dl). All seven patients had hyperparathyroidism with an average of 733 pg/ml (range from 113 pg/ml to 3193 pg/ml). En bloc resection was performed in two patients with neighboring structure invasion, and four patients with complete tumor capsules underwent tumor resection with limited resection of the thyroid gland. Postoperative adjuvant radiotherapy appeared unsuccessful for local recurrence.

**Conclusion:**

High calcium, high PTH, parathyroid occupation by ultrasound, and intraoperative invasion should be considered to have the possibility of parathyroid cancer. Open surgery is recommended and protecting tumor integration is the elementary surgery principle. The initial surgical extent should be decided by the invasion of the tumor. When PC has a local recurrence, the debulking surgery and adjuvant radiotherapy are always fake.

## 1. Introduction

Parathyroid carcinoma (PC) is a rare malignant neoplasm involving the parathyroid gland and one of the rarest causes of primary hyperparathyroidism (PHPT), which was first described by Sainton & Millot in 1933 [1]. Hypercalcemia is the most obvious and severe symptom of PC, the major contributor to poor quality of life and mortality in PC patients, and can lead to kidney stones, fatigue, bone pain, etc. [2]. However, few reported clinical cases show that nonfunctioning parathyroid carcinoma is in the absence of hypercalcemia, although routine cervical ultrasound for anatomical localization might be suggestive of the diagnosis [3, 4]. Until now, features and diagnosis of PC still seem to be confusing in the clinic. The recurrence rate of PC is as high as 65%. And the10-year survival rate is reported from 49%-87%, as reported by various studies [3, 5, 6]. At present, the major treatment for PC is surgery, as some experts have suggested en bloc resection is the preferred operation [1, 5, 7, 8]. However, there is still no agreement on the optimal extent of the initial surgery, for limited clinical reports focusing on the operation type and the uncertain correlation between surgical extent and prognosis.

The article "The Clinical Features and Treatment Strategy of Parathyroid Cancer: A Retrospective Analysis" was published in 2022. Journal: Biomed Res Int.

We report our experience with PC which includes three cases of nonfunctioning and four cases of functioning PC and contrast the features of these two varieties of the same disease. And we conclude their different types of operation and prognosis, trying to explore the more reasonable treatment of PC.

## 2. Materials and Methods

### 2.1. The Patients

We retrospectively analyze the clinical data of seven patients with PC in Shanxi Bethune Hospital, the Third Hospital of the Shanxi Medical University of China, who underwent the initial surgery from 2014 to 2021. Included patients underwent initial surgery and were clearly diagnosed with PC by histology of their tissue sections based on histopathologic criteria. In each case, the medical records were complete, including clinical manifestations, preoperative diagnosis, preoperative laboratory examinations (including PTH level, serum calcium level, and alkaline phosphatase measured in the peripheral blood), surgical type, histology, and diagnosis documented. Each patient is followed up until March 2022 by outpatient or phone. Most of their PTH and Calcium level was tested repeatedly after the initial surgery to realize postoperative recurrence. Some patients also underwent ultrasound or SPECT-CT during follow-up. Exclusion criteria included patients without follow-up and patients with incomplete records. Written informed consent including treatment, medical records, and all clinical data of patients was obtained from all participants. The study has been reviewed and approved by Shanxi Bethune Hospital Institutional Review Board.

### 2.2. Treatment

For the primary tumor, three types of surgical resection were performed, including type 1 which is the en bloc resection (tumor resection with ipsilateral thyroid lobectomy or the ipsilateral and the isthmus of the thyroid lobectomy), type 2 which is the resection of the tumor and the limited surrounding thyroid tissue, and type 3 which is the tumor resection only by the endoscopy. PC is difficult to be diagnosed before the surgery, thus the surgical type is divided by the extent of the invasion shown in the surgery process. Most of our PC patients that had the tumor with complete capsule underwent type 2 surgery. Patients with tumors invading the neighboring structure or close to the neighboring structure, such as muscles, recurrent nerve or esophageal wall underwent type 1 surgery. Type 3 surgery was only found in patient 5. The ultrasound of all patients did not show any lymph nodes suspicious of metastasis. For the lymph node dissection, four patients did not take lymph node dissection for the invisible enlarged lymph nodes during detection; two patients had central compartment dissection with the enlarged lymph nodes detected in surgery which showed no metastasis by histopathology. Postoperative external radiation therapy (RT) was performed on a local recurrent patient (patient 5). Systemic chemotherapy plus preoperative RT was not performed on any of the patients included.

The article "The Clinical Features and Treatment Strategy of Parathyroid Cancer: A Retrospective Analysis" was published in 2022. Journal: Biomed Res Int.

## 3. Results

### 3.1. Patient Characteristics

The clinical features, tumor characteristics, and initial operation are summarized in Table 1.

In our study, there are seven patients diagnosed with PC after the initial operation. Four of seven patients were men and the other three were female, whose average age was 55 (ranging from 39 yrs to 70 yrs). Four patients (patients 1, 3, 5, 6–57%) were diagnosed or suspected of parathyroid occupation. Between them, two patients had multiple bone fractures, one patient had kidney involvement, and one patient was present with abdominal distension. The other three patients (patients 2, 4, 5–43%) were diagnosed with thyroid tumor, in which patient 4 mainly manifested hematoma of the neck (Figures 1 and 2). In all seven patients, only one patient (patient 6) had hoarseness with 2 years course before treatment. The other six patients only had a short course before finding occupation in the ENT department.

Marked hypercalcemia, which was revealed to be an average of 13.9 mg/dl (ranging from 11.8 mg/dl to 15.8 mg/dl), was observed in four patients (57%). The others' serum calcium levels were in the normal range with an average of 9.9 mg/mg/dl (ranging from 8.6 mg/dl to 10.8 mg/dl). Similarly, increased alkaline phosphatase, which was revealed to be an average of 1086.7 IU/L (ranging from 176.8 IU/L to 2733.8 IU/L), was observed in four patients (57%). And the others' alkaline phosphatase level was in the normal range with an average of 75 IU/L (ranging from 54 IU/L to 97.3 IU/L). Besides, all seven patients are significantly found to have hyperparathyroidism. The average maximum diameter of the tumor was 50 mm (17–50 mm) in histological specimens. The tumors of five patients had capsular invasiveness by histology, and the tumors of two patients had neighboring soft tissue invasion. Patient 7 had conglutination with the esophagus and recurrent laryngeal nerve.

The article "The Clinical Features and Treatment Strategy of Parathyroid Cancer: A Retrospective Analysis" was published in 2022. Journal: Biomed Res Int.

### 3.2. Initial Surgery and Follow-Up

En bloc resection was performed in two patients, and four patients underwent tumor resection with the limited thyroid gland. Only one patient underwent endoscopic surgery in General Surgery Department. Patient 4 of our study is a special case who presented with a hematoma of the neck (Figures 1 and 2). During the initial surgery, we observed that the tumor with the neighboring thyroid had a complete capsule, but had a hematoma that might cause by the neighboring thyroid vascular invasion. The big hematoma had the adhesion with neighboring muscles and carotid sheath, with no clear evidence of invasion of these structures. Thus, this patient underwent the en bloc resection with the isthmus of the ipsilateral thyroid gland. Lymph node and distant metastases were not found preoperatively in all patients who underwent initial surgery. Ipsilateral central node dissection dissections were performed in two patients.

The average follow-up period was 36 months following the initial treatment. Six patients did not have postoperative hypercalcemia or hyperparathyroidism, and currently have no evidence of the recurrence. Patient 5 who underwent endoscopic surgery immediately got local recurrence in the right lobe of the thyroid after 8 months (Figure 3). And then underwent the resection with the right lobe of the thyroid, the isthmus of the ipsilateral thyroid, and ipsilateral central node dissection. After the remedial operation, that patient performed postoperative adjuvant radiotherapy. 1 year later, with chest wall recurrence happening unavoidably, patient 5 undertook the tumor resection of the chest wall (Figure 4). In the second year, this patient had distant metastases and used drugs to control hypercalcemia.

## 4. Discussion

### 4.1. Diagnosis and Features

PC is an exceedingly rare disease, which accounts for less than 1% of presentations of primary hyperparathyroidism, although with an exponential increase in the number of patients presenting with PC [7, 9]. Most PC is clinically silent and not diagnosed preoperatively or intraoperatively [10]. And suspicion signs may include severe bone and kidney involvement, palpable neck mass, hoarseness, or palpable, enlarged neck lymph nodes. Laboratory findings include markedly increased PTH levels (>5 times above normal levels) and serum calcium concentrations (usually exceeding14–15 mg/dl) [5, 11]. However, it is still very difficult to diagnose PC before surgery, because the symptoms of PC are not typical [7, 12, 13]. Some patients only presented with thyroid or parathyroid nodules. Even, a PC patient showed thyroid occupation and neck hematomas, which present as acute petechiae in the neck and the hematomas of the oropharynx (Figures 1 and 2). Due to the insidious symptoms, the preoperative diagnosis for PC is difficult. At present, the diagnosis of PC requires a comprehensive consideration of blood calcium, PTH, ultrasound, and intraoperative invasion.

The article "The Clinical Features and Treatment Strategy of Parathyroid Cancer: A Retrospective Analysis" was published in 2022. Journal: Biomed Res Int.

Patients with serum calcium levels greater than 1.15 times the upper normal limit or 14 mg/dl can be suspected to have PC [11, 14]. Besides, a higher calcium level at recurrence and the use of a high number of calcium-lowering medications after the diagnosis of cancer increased mortality [14]. PC is generally hyperfunctioning, but less than 10% of patients have no clinical manifestations of hyperparathyroidism [7, 11, 13]. In our study, three of seven patients are at the normal level of serum calcium with an average of 9.9 mg/dl (ranging from 8.6 mg/dl to 10.8 mg/dl). The other four patients are in a higher level of serum calcium with an average of 13.9 mg/dl. We do agree that the possibility of having a PC should be considered for patients with parathyroid or thyroid occupation and a higher calcium level greater than 14 mg/dl. However, blood calcium in some PC patients is within the normal range, and it is very difficult for such patients to diagnose as PC. And those patients take up to 43% of all PC patients in our study. Thus, calcium level cannot be the only evidence for the diagnosis of PC. Alkaline Phosphatase (ALP) levels were presented in 20 papers, four of which showed significantly higher in PC patients [15]. We also focus on the ALP of these PC patients included in our study. We found that not all PC patients had an increased ALP level, which is the same as calcium. Thus, we think that there are some PC patients with normal calcium and ALP. For these patients, other features should be imperative, such as PTH and intraoperative invasion.

Our study showed that PTH may be a better suggestive index rather than calcium. Patients with serum PTH level which is greater than three times the upper normal limit is highly thought to be PC [11]. In our study, all cases both functioning and nonfunctioning had a high level of PTH with an average of 733 pg/ml, which ranges from 113 pg/ml to 3193 pg/ml(1.6 to 45.6 times higher than the normal). PTH of functioning PC is far more increased than the normal limit and even much more than patients with parathyroid adenoma which was reported to be 136 ± 6 pg/ml(1.9 times of normal range) [16]. Also in our study, patients with nonfunctioning PC have an average PTH level of 173.5 pg/ml (2.5 times of normal range), which is higher than patients with parathyroid adenoma. Besides, PTH is also used in the operation and follow-up of PC. As reported, high serum PTH is also predictive of the occurrence of PC, which might be an important index in the follow-up PC [11]. But intraoperative PTH monitoring is still under debate [17].

The article "The Clinical Features and Treatment Strategy of Parathyroid Cancer: A Retrospective Analysis" was published in 2022. Journal: Biomed Res Int.

Palpable neck mass is suspected to be PC, and a high index of suspicion is warranted for lesions larger than 3 cm or presenting [18]. In our study, the tumor is in an average size of 3 cm, ranging from 1.7 cm to 5 cm. And we find that the tumor size is not related to the tumor function. Most PC is not diagnosed intraoperatively with many tumors being diagnosed postoperatively with the benefit of immunohistochemistry. But operative findings of local invasion, a very large tumor or thick adherent capsule, and gland weight >2000 mg can be the criteria that raise the intraoperative suspicion of PC [10]. The invasion of recurrent nerve or esophageal wall and/or the presence of lymph node metastases have the greatest predictive value [4, 5]. Studies also found that nonfunctioning PC may be more aggressive than their functioning counterpart [3]. In our study, most patients did not show intraoperative invasion, while only two patients showed a correlation with neighboring structures. Especially, patient 7 showed esophagus and recurrent laryngeal nerve invasion in operation. And we also found that the intraoperative invasion was not connected to the level of PTH or calcium in PC patients. Not all PC patients had neighboring invasion but we agree that intraoperative invasion can be a vital clue for PC.

Some studies pointed out that a routine cervical ultrasound for anatomical localization might be suggestive of the diagnosis [3]. While the ultrasound of PC is still controversial, some others suggest scintigraphy might be better [8]. On ultrasound, PC may have ill-defined margins and signs of invasion of surrounding structures, as well as lymph node metastases [5]. A study suggested a high positive predictive value for cancer was identified for infiltration and calcification, while a high negative predictive value was found for the absence of suspicious vascularity, a thick capsule, and inhomogeneity [19]. Our study shows that a routine cervical ultrasound can sensitively find the occupation of the mass or nodes in the thyroid or parathyroid, but does not precisely distinguish the accurate origination and the malignancy, because ultrasound images are not typical. In our study, six out of seven patients presented with clear margins and regular morphology in cervical ultrasound. Only one patient's ultrasound showed unclear margins and irregular morphology. However, a repeat cervical ultrasound is useful for the recurrence in the follow-up [20]. Our patient 5 found local recurrence and chest wall metastasis by ultrasound. At present, partial experts still think there are no trials to prove the best imaging modalities, but recommended that a repeat neck ultrasound can be done in 3–6 months in follow-up [1].

The article "The Clinical Features and Treatment Strategy of Parathyroid Cancer: A Retrospective Analysis" was published in 2022. Journal: Biomed Res Int.

### 4.2. Initial Surgery

PC is reported to have high recurrence rates after the initial surgery, which is always a barrier to the cure of PC patients. Thus, that makes PC a disease difficult to treat. Harari et al. reported that 49% of PC patients had recurrence after initial cancer operation and had a frequent need for reoperations in the follow-up period of 43 years [14]. Another study shows that as many as 65% of patients with parathyroid carcinomas will have cervical recurrence after the initial operation [3]. In a cohort study, 12 of the 41 patients (29%) presented with or developed recurrent disease, either at diagnosis or after a median follow-up period of 6.5 years [11]. The high recurrence rate is mostly due to the invasion of the tumor. Most studies support that the invasion of recurrent nerve or esophageal wall and/or the presence of lymph node metastases has the greatest predictive value in recurrence [5, 7, 21]. Whether the extent of operation was associated with mortality or was it associated with the number of recurrences or neck dissections required is explored by many studies [14]. Most studies showed that, concerning the management of PC, the first operation offers the best chance of cure [10, 13]. However, the extent of the initial surgery of PC is still in dispute.

With the continued improvements in parathyroid imaging techniques, minimally invasive parathyroidectomy is rapidly becoming the procedure of choice in patients with benign parathyroid tumors [16]. The introduction of minimally invasive parathyroidectomy techniques has meant that most parathyroid surgery can now be performed on an ambulatory basis through a 2 cm mini incision [10]. But as to the PC patients, we think the minimally invasive parathyroidectomy techniques might not be the same. In our study, a PC patient with a solid occupation of 2.6 × 1.5 cm in the right parathyroid showed unclear margins and irregular morphology by ultrasound preoperatively. That patient underwent right parathyroid resection by endoscopy. However, that patient immediately had local recurrence 8 months after the initial surgery and then, continued to take enlarged thyroid resection with selective central node dissection and adjuvant radiotherapy. After 1 year of the initial surgery, that patient had a chest wall metastasis, right in the path of the endoscopy. For that tumor had a complete capsule by detection, we think the recurrence may be due to the intraoperative tumor rupture caused by the limited operating skills and careless operation during endoscopic surgery. And the chest wall recurrence should be the scattered tumor cells in the surgical path when got the ruptured tumor out (Figure 4). As reported, protecting tumor integration is the most elementary surgery principle of PC [22]. Intraoperative tumor rupture is the first factor that predicts the recurrence of PC [5]. Rupture of the tumor capsule during the primary operation, followed by frequent local recurrences, has been described [3]. A careful operative technique during the primary operation is essential for preventing seeding of the operative field with malignant cells. Thus, we support that endoscopic surgery is not recommended if cannot guarantee a complete capsule or remove the whole tumor.

The article "The Clinical Features and Treatment Strategy of Parathyroid Cancer: A Retrospective Analysis" was published in 2022. Journal: Biomed Res Int.

At present, most PC patients are recommended to open surgery, aiming to resect the tumor with the complete capsule. But the surgery extent is still under debate. The most commonly performed resections are simple tumor excision (parathyroidectomy) and en bloc resection [9]. The local excision alone is not recommended at present [10, 13, 14], because not all the tumors had the complete capsule. The local excision alone might result in a significantly higher risk of failing to achieve complete resection of the primary cancer lesion, which might associate with higher rates of local-regional recurrence and lower disease-free survival [18]. An en-bloc resection is a suggestive surgery for PC, with requires, as a minimum, ipsilateral hemithyroidectomy [10]. The removal of the ipsilateral thyroid may be the easiest and safest way forward whenever the parathyroid touches the thyroid plane [18]. But this surgery extent can cause some patients to get hypothyroidism, and some patients have to take Euthyrox for the rest of their life. Also in a study, the en bloc resection is found not associated with improved survival [9]. We support that the surgical extent should be divided by the extent of the invasion by tumor. For the tumor with a complete capsule, parathyroidectomy with the limited neighboring thyroid gland is sufficient for PC patients. Margin involvement and intraoperative tumor rupture are potentially confounding factors in the recurrence of PC. It is well-established that disease-positive resection margins are associated with increased local recurrence rates [5, 10]. Parathyroidectomy with a limited neighboring thyroid gland can also achieve an uninvolved margin. In our study, the average follow-up time is 35months (ranging from 10–90months). During the follow-up time, four patients with tumors and limited resection of the neighboring thyroid resection did not have a recurrence. But for the tumor has invaded the neighboring structure, such as muscles, recurrent nerve, or esophageal wall, the en bloc resection may be performed more frequently and can achieve an uninvolved margin better.

The article "The Clinical Features and Treatment Strategy of Parathyroid Cancer: A Retrospective Analysis" was published in 2022. Journal: Biomed Res Int.

There is some controversy about the initial surgical management of the neck lymph nodes. Some investigators suggest an en bloc removal of the primary lesion should include ipsilateral radical neck dissections with special attention to the nodes in the tracheoesophageal groove [3]. Because level VI dissection does not impose a significant risk to the patient, it should be an integral part of the procedure [18, 23]. While, it has been suggested that since metastasis to regional lymph nodes is rare and occurs late in the disease, radical neck dissection should not be considered unless the nodes are grossly involved [3, 9]. Some experts suggest a prophylactic selective ipsilateral central node dissection is recommended [11]. Concerning the treatment of lymph node metastases, the majority of authors recommend ipsilateral central cervical lymph node dissection as part of initial surgery, although its implementation in surgical practice is limited [5]. But a study found that there are no data to support this as less than 10% have nodal involvement [10]. Another study also showed that lymph nodes were not found preoperatively in 11 patients of 12 who underwent initial surgery for PC [24]. In our study, all seven patients did not show preoperative lymph node involvement. Between these patients, 2 patients underwent DI. Comparing D0 and D1 in our study, local recurrence appears to be more associated with intraoperative tumor rupture. Besides, PC is commonly diagnosed after surgery for primary hyperparathyroidism. Lymph node dissection is also controversial in patients whose intraoperative freezing section does not get a definite diagnosis. Thus, appropriate selective node dissection of involved lymph node compartments is recommended when there has clinical evidence of nodal involvement [9].

### 4.3. Treatment of Recurrence

The malignancy of PC is high, but the prognosis and the overall survival are still uncertain for the small number of cases. The analysis included data from 37 patients who received a primary operation or treatment for PC. The data covered a period of 43 years. The study showed that 48.7% of patients had died and the median overall survival was 14.3 years from diagnosis [14]. Another study observed a 10-year disease-free survival of 79% [11]. The prognostic related factors of PC patients are currently under study. Lymph node or distant metastases, the number of recurrences, high calcium level at recurrence, and use of a high number of calcium-lowering medications might be factors independently associated with increased mortality [14]. Besides, disease-specific death of PC is related to intraoperative tumor rupture and distant disease relapse [5].

The article "The Clinical Features and Treatment Strategy of Parathyroid Cancer: A Retrospective Analysis" was published in 2022. Journal: Biomed Res Int.

A study sorted out the causes of death in detail and find that patients with functioning PC generally die from complications of hypercalcemia, thus, control of hypercalcemia is the long-term goal in their cases. For patients with local recurrences, hypercalcemia is best treated with excision surgery [3, 13]. Excision of surgical accessible sites of metastases, bone, lung, and liver is recommended [10]. Kawagishi et al. reports a case of debulking surgery for functional pleural dissemination of parathyroid carcinoma. In this case, the debulking surgery decreased temporarily activities of the PTH level [25]. While in our study, patient 5 had a local recurrence and chest wall metastasis, but the second debulking surgery failed with the distant metastasis in the end. Thus, debulking surgery is most often palliative and seldom curative [3].

There is some doubt if these patients would have better local control when they were offered adjuvant radiotherapy [8]. Some studies supported that adjuvant radiotherapy may improve local control and limit the occurrence of local relapse [26]. But other studies show that external beam radiotherapy is of no demonstrated benefit for them [10, 23]. In a cohort, 4 of the 5 patients who received adjuvant radiotherapy experienced tumor recurrence, of whom 3 died [11]. 11 patients in the current study also showed no significant differences between the groups of patients with or without postoperative adjuvant radiotherapy [24]. Another study also contrasts that radiotherapy may result in a lower risk of local regional disease progression and improved cause-specific survival [27]. In our experience with patient 5, adjuvant radiotherapy seems to have no significant effect. In these patients with advanced disease and distant metastasis, multimodality treatment rarely achieves a cure. Systemic therapies, sometimes in conjunction with external beam radiation therapy and conventional chemotherapy, have failed to demonstrate efficacy [1, 12]. Some experts point out that immunotherapy may hold promise for adjuvant treatment of PC [11]. But additional research to better understand PC, tumorigenesis, and explore the use of immunotherapy or other targeted therapies is still needed [1].

## 5. Conclusions

In conclusion, PC is a rare and thorny disease, which is clinically silent and diagnosed with difficultly. Our study focused on the features, initial surgery extent, and the treatment of recurrence, and tried to improve the preoperative diagnosis possibility and reduce the recurrence. Our study showed that calcium level is unreliable for parts of patients, ultrasound is nonspecific, and invasion of neighboring structures does not always appear. But, we found that PTH is reliable higher than 14 pg/ml can be an imperative and reliable clue for PC. Besides, comprehensive consideration of ultrasound and intraoperative invasion can improve the diagnosis preoperatively. The initial surgery of PC is vital. Endoscopic surgery is not recommended for PC patients when cannot make sure the tumor is integrated. We support that the surgical extent should be divided by the extent of the invasion by tumor. For the tumor with a complete capsule, parathyroidectomy with the limited neighboring thyroid gland is sufficient. En bloc resection may be performed better in patients with local invasion. Also, we found that most of our patients did not have lymph node metastasis, thus appropriate selective node dissection of involved lymph node compartments is recommended when there has clinical evidence of nodal involvement. When PC has a local recurrence, the debulking surgery and adjuvant radiotherapy are always fake.

The article "The Clinical Features and Treatment Strategy of Parathyroid Cancer: A Retrospective Analysis" was published in 2022. Journal: Biomed Res Int.

## Figures and Tables

**Figure 1:** Patient 4 mainly manifested the hematoma of the neck.

**Figure 2:** The CT of the neck in patient 4, showing occupation of the right thyroid lobe.

**Figure 3:** This is the thyroid ultrasound of patient 5 who underwent endoscopic surgery 8 months after the initial surgery. The ultrasound showed a local recurrence in the right lobe of the thyroid, with unclear margins and irregular shape.

**Figure 4:** This is the chest wall ultrasound of patient 5. That showed a chest wall recurrence a year after the initial surgery, presented with occupation and irregular margins.

**Table 1:** Characteristics of Patients with Parathyroid Carcinoma.

Patient	Age[yr.]/sex	Clinical manifestation	Initial calcium[mg/dl]	PTH[pg/ml]	Alkaline Phosphatase[IU/L]	Ultrasound/CT	The extent of disease at the initial operation	Invasion saw in operation	Follow-up[month]	Recurrence/metastases
1	46/F	Parathyroid nodule for 1 month	8.6	113	73.8	Left parathyroid nodules; inhomogeneity; clear margins;2.1 × 1.2 cm	Tumor resection with limited resection of the neighboring thyroid gland	N	90	N
2	50/F	Thyroid nodule for 2 months	13.4	804.6	823.3	Solid nodules in the right lobe of the thyroid; clear margins; regular morphology; 4.8 × 2.4 cm	Tumor resection with limited resection of the neighboring thyroid gland; the ipsilateral central node dissection	N	36	N
3	39/F	Urinary stones and hydronephrosis; multiple bone fractures; parathyroid occupation for 10 days	15.8	3192	2733.8	A solid nodule in the lower left parathyroid; clear margins; Regular morphology; 3.9 × 1.5 cm	Tumor resection with limited resection of the neighboring thyroid gland	N	30	N
4	70/M	Hematoma of the neck for 5 days with thyroid occupation	10.32	273.1	54	The solid nodule in the middle of the right thyroid; clear margins; regular morphology; 4.4 × 3 × 3.3 cm	Tumor resection with the right lobe and the isthmus of the ipsilateral thyroid gland; ipsilateral central node dissection	Adhesion with neighboring thyroid gland; neighboring muscles; carotid sheath	20	N
5	64/M	Weakness in both lower extremities for 1 year; Abdominal distension for 1 month; Parathyroid occupation for 10 days	14.44	189	613	Solid occupation of the right parathyroid; unclear margins; irregular morphology; 2.6 × 1.5 cm	Endoscopic right parathyroid resection	N	48	Local recurrence in 8 months after surgery 1 year after surgery, chest wall recurrence 2 years after surgery, distant metastases
6	56/M	Parathyroid occupation for 10 days	10.8	134.5	97.3	A solid nodule of the right parathyroid; inhomogeneity; Clear margins; regular morphology; 1.7 × 1.0 cm	Tumor resection with limited resection of the neighboring thyroid gland	N	12	N
7	64/M	Thyroid occupation for 2 years;	11.8	425	176.8	A solid occupation in the left lobe of the thyroid; clear margins; regular morphology; 5 × 3.1 cm	Tumor resection with ipsilateral hemithyroidectomy	Neighboring thyroid gland; esophagus; recurrent laryngeal nerve	10	N

The article "The Clinical Features and Treatment Strategy of Parathyroid Cancer: A Retrospective Analysis" was published in 2022. Journal: Biomed Res Int.

## Data Availability

All data are in within the article.
